RETRACTED

# miR-190a-3p Promotes Proliferation and Migration in Glioma Cells via YOD1

**DOI:** 10.1155/2021/3957738

**Published:** 2021-09-04

**Authors:** Lili Zhou, Lingzhi Li, Yan Chen, Chun Chen, Zhongwen Zhi, Luxia Yan, Yuqian Wang, Bing Liu, Qijin Zhai

**Affiliations:** ^1^Department of Neurology, The Affiliated Huai'an Hospital of Xuzhou Medical University, Huai'an, 223002 Jiangsu, China; ^2^Department of ICU in Emergency Center, The Affiliated Huai'an Hospital of Xuzhou Medical University, Huai'an, 223002 Jiangsu, China; ^3^Department of Neurology, Siyang Hospital of Traditional Chinese Medicine, Siyang, 223700 Jiangsu, China

## Abstract

**Introduction:**

To investigate the function of miR-190a-3p on the proliferation and migration of glioma.

**Methods:**

Twenty glioma samples and 6 normal brain tissue samples were collected. Normal human glial cell line HEB and glioma cell lines were used for the experiments. We then used TargetScan to predict the target genes of miR-190a-3p. Dual-luciferase reporter assay was also used to validate.

**Results:**

Combined with dual-luciferase reporter experiment, we finally verified that YOD1 was the aim, and it was low-expressed in glioma. Besides, a series of mechanism experiments then proved that miR-190a-3p negatively regulates YOD1 expression.

**Conclusions:**

Our research was the first to demonstrate the promoting function of miR-190a-3p in the proliferation and migration of glioma and provided new views for the treatment of glioma. miR-190a-3p was expected to be a new target for molecular therapy of glioma.

## 1. Introduction

Glioma is one of the most usual primary intracranial tumors, accounting for nearly 50% of all primary intracranial tumors [1]. It is characterized by high morbidity, mortality, and poor prognosis [2]. According to the degree of malignancy, glioma can be divided into astrocytoma, oligodendroglioma, stromal oligodendroglioma, and glioblastoma. Patients with highly malignant glioblastoma multiforme have a median survival time less than one year. Glioma is highly aggressive which shows invasive growth and has an unclear boundary with healthy brain tissue [3]. At present, the therapy of glioma mainly rely on the surgery-assisted radiotherapy and chemotherapy, and the patients who suffer from these treatments often have poor prognosis and are very prone to relapse [4]. The occurrence and development of glioma are a comprehensive process involving multiple factors, genes, and molecules. Based on the current status of glioma, the treatment and survival of patients, researches on the pathogenesis of glioma are urgently needed to lay the foundation for the subsequent study of glioma and to provide new points for the therapy of glioma.

miRNAs are series of 20 to 22 nt RNAs without protein-coding function. miRNAs regulate the mRNA expression via combining with the target mRNA [5]. They participate in a series of biological processes, for example, cell propagation and differentiation, stress, and apoptosis, and therefore have important significance in tumor research [6]. Ciafrè et al. analyzed 245 miRNAs in 9 pairs of human glioma tissues and 10 glioma cell lines. They found that 20 miRNAs are expressed differently in glioma, of which 9 miRNA are upregulated; 11 miRNA are downregulated [7]. Liu et al. analyzed medulloblastoma tissue through high-throughput microarray technology and found that miR-113, miR-99a, miR-102, and miR-109b are significantly increased, whereas miR-216, miR-29a, miR-128a, miR-29c, and miR-128-5p are significantly reduced [8]. With the progress of miRNA research, more and more scholars have discovered that miRNAs may be involved in regulating malignant progression, angiogenesis, growth, recurrence, and migration of glioma [9–12].

miR-190 has two primary mature forms, including miR-190a-5p and miR-190a-3p [13]. It is well known that miR-190a-5p plays an essential part in various diseases, especially in malignant tumors. According to the reports, miR-190a-5p acts a dual role in different cancers, for instance, miR-190a-5p is increased in bladder cancer and gastric cancer, while it is decreased in rectal cancer and liver cancer [14–16]. However, the function of miR-190a-3p in various diseases is still poorly understood.

RETRACTED

YOD1 is a well-known deubiquitinating enzyme, and it is highly conserved that can cleave ubiquitin residues of ubiquitinated proteins, but its function has not been determined in mammalian cells yet [17]. Ubiquitination and deubiquitination of proteins control many biological processes, such as cell cycle, transcriptional activation, and signal transduction, and are closely associated with the tumorigenesis [18]. Deubiquitination is known to stabilize tumor suppressor genes and thus inhibit the occurrence and progression of tumors [19]. In the current research, we confirmed that miR-190a-3p promoted the proliferation and migration of glioma by inhibiting the expression of YOD1, which provided new ideas for the therapy of glioma.

## 2. Materials and Methods

### 2.1. Clinical Specimens

20 glioma samples and 6 normal brain tissue samples were collected from The Affiliated Huai'an Hospital of Xuzhou Medical University during 2019-2020. The 20 glioma tissue samples were graded according to the WHO glioma grading standard. Tissues were frozen in liquid nitrogen until further RNA extraction. This study had been ratified by the Ethics Committee of The Affiliated Huai'an Hospital of Xuzhou Medical University. All patients or their relatives had signed informed consents in advance.

RETRACTED

### 2.2. Cell Culture

Normal human glial cell line HEB and glioma cell lines T98G, U87, SHG44, and U251 were bought from Tongpai Biotechnology (Shanghai, China). DMEM with high glucose and sodium glutamate (Hyclone, GE, Marlborough, USA), added with 10% FBS (Gibco, Invitrogen, California, USA) and 1% antibiotic mixture (Sigma-Aldrich, St. Louis, USA), was applied to culture cells. All cells were cultivated in a 37°C incubator (Panasonic, Osaka, Japan) containing 5% CO_2_.

### 2.3. Cell Transfection

The miR-190a-3p inhibitor expression plasmid (pGCMV-EGFP-miR-190a-3p inhibitor), shYOD1 expression plasmid (pGPU6-Neo-shYOD1), and their corresponding negative control plasmid were constructed by GenePharma (Shanghai, China). The logarithmic phase U87 and U521 cells were inoculated in plates overnight to 80% confluence, then change to serum-free DMEM. The mixture of Lipo3000 transfection regents (Sangon Biotech, Shanghai, China) and miR-190a-3p inhibitor expression plasmid, shYOD1 expression plasmid, and NC plasmid was prepared by serum-free DMEM and then added into the wells. 4 h later, the normal DMEM was changed and the subsequent experiments were carried out after 24 h of cultivation. Transfection efficiency of miR-190a-3p inhibitor was detected by the GFP under the microscope. Cell lines stably transfected with YOD1 shRNA were screened by neomycin.

### 2.4. Real-Time Quantitative PCR

Total RNA was extracted by using a commercial extraction kit (Biomarker, Beijing, China) that followed the instructions in the product manual. The SYBR Green RT-qPCR kit was obtained from Biosharp (Hefei, China), and the SLAN-96S Real-time PCR System (HongShi, China) was used to examine the level of miR-190a-3p and YOD1. U6 and *β*-actin were internal references. A 2^−*ΔΔ*Ct^ method was applied for relative quantitative analysis. All primers used are listed in Table 1.

### 2.5. Cell Proliferation

U87 and U251 cells were first inoculated in cell culture plates and grown to 80% confluence, respectively, then added 10 μl CCK-8 reagent (Sangon Biotech, Shanghai, China) per well, and continued to cultivate cells for another 4 h. Finally, OD_450_ was measured using a microplate reader (Synergy H1, USA) to determine the cell viability.

### 2.6. Colony Formation Assay

The logarithmic growth phased U87 and U251 cells were digested into single cells and inoculated in a Petri dish with 200 cells per well, then cultured cells for 2-3 weeks until visible colonies appeared. The supernatant was discarded, washed with PBS twice, then treated with fixative for 15 min, stained with Giemsa for 30 min, and finally, rinsed with PBS for at least five times. The number of clones was calculated under the microscope.

RETRACTED

### 2.7. Wound Healing Assay

Glioma cells introduced with miR-190a-3p or NC inhibitor were inoculated in a 6-well plate until grown to 90% confluence. Use a sterile tip to cause a wound line in each well, then record the wound healing under the microscope at 0 h and 48 h after the operation. The wound healing degree was calculated by software.

### 2.8. Transwell Migration and Invasion Assay

Cells treated with miR-190a-3p or NC inhibitor were digested and seeded in the Transwell chamber without Matrigel (Millipore, USA). After 24 h, cells in the lower chamber were immobilized with aldehyde fixative for 30 min and then stained with 0.1% crystal violet, and photos were shot with the microscope. The procedure for the invasion experiment is the same as above, except that the Transwell chamber used for the invasion experiment was covered with Matrigel on the upper side.

### 2.9. Western Blot

Preparing cell lysates with RIPA Buffer (Solarbio, China) for the first, the protein content was analyzed with the BCA Kit (Solarbio, China). SDS-PAGE was conducted and then transferred the separated protein to the PVDF film. Blocked with BSA, the film was treated with the primary antibody and secondary antibody in sequence and finally developed with enhanced chemiluminescence reagent ECL (PE0010, Solarbio, China). All antibodies used in this article were purchased from Abcam (Cambridge, MA).

### 2.10. TUNEL Assay

Cells were first inoculated in 24-well plates and grown until 80% confluence. Discarding the upper medium, the cells were fixed in turn with fixative and permeated with operating instructions of the TUNEL reaction kit (Beyotime, China). Then, add DAPI dye for staining cells and recording with a fluorescence microscope at a wavelength of 490 nm; the apoptotic cells represented green fluorescence. Using software to calculate the apoptosis rate.

### 2.11. Dual-Luciferase Reporter Assay

YOD1 was screened to be the target of miR-190a-3p that related to glioma by using TargetScan 7.2 software. The wild-type and mutant 3′UTR of YOD1 were synthesized and inserted into the pmirGLO dual-luciferase reporter vector (Biovector, China). miR-190a-3p/NC mimics and the vector were cotransfected to glioma cell lines with Lipo3000 Reagent (Invitrogen, CA, USA). Luciferase activity of cells was detected after 48 h.

### 2.12. Statistical Analysis

The data were expressed as the mean ± standard deviation (SD) of three parallel experiments. Using SPSS 23.0 for data statistics, GraphPad was also used for survival curves. *p* < 0.05 was considered statistically significant.

RETRACTED

## 3. Results

### 3.1. miR-190a-3p Is High-Expressed in Glioma

Firstly, we checked the level of miR-190a-3p in both glioma tissues and cell lines to explore the relationship between the miR-190a-3p and the glioma. As seen in Figure 1(a), the level of miR-190a-3p in glioma tissues was much higher. Furthermore, miR-190a-3p was also higher in grade III+IV glioma than that in grade I+II (Figure 1(b)). By analyzing the miR-190a-3p level and the overall survival rate of included clinical samples, we found that the survival rate was lower in samples with the high-level miR-190a-3p, as shown in Figure 1(c). Next, we tested the miR-190a-3p level in a series of glioma cell lines. It was obvious that miR-190a-3p was low-expressed in HEB cells but was highly expressed in T98G, U87, SHG44, and U251 cell lines (Figure 1(d)). Besides, we designed and transfected miR-190a-3p inhibitor into U87 and U251 cell lines to further seek the effect of miR-190a-3p in glioma (Figure 1(f)). Herein, GFP was used to verify the transfection efficiency of miR-190a-3p inhibitor (Figure 1(e)).

### 3.2. Suppression of miR-190a-3p Inhibits the Proliferation of Glioma and Promotes Its Apoptosis

Through CCK-8 and colony formation experiment, we found that the cell viability of U87 and U251 decreased significantly after adding the miR-190a-3p inhibitor (Figure 2(a)), and the number of colonies was also considerably reduced (Figure 2(b)), which indicated that suppression of miR-190a-3p restrains the propagation of glioma cells. Next, we studied the apoptosis of glioma cells after introducing miR-190a-3p. The results of TUNEL showed that the apoptosis of cells was increased after the addition of miR-190a-3p inhibitor; at least 50% of cells had undergone apoptosis (Figure 2(c)). Moreover, the expression of a few proteins that were related to apoptosis was examined. It was shown in Figure 2(d) that the level of Bax and cleaved caspase-3/9 was increased, whereas Bcl-2 was decreased.

### 3.3. Suppression of miR-190a-3p Inhibits the Progression of Glioma

In order to investigate the effect of suppression of miR-190a-3p on the progression of glioma, wound healing and Transwell assays were conducted. It could be seen that the wounds were caused after 48 h, and the wounds of U87 and U251 cells gradually healed (Figure 3(a)). Moreover, as shown in Figures 3(b) and 3(c), introducing miR-190a-3p inhibitor obviously impeded the migration and invasion of cells. Furthermore, after miR-190a-3p was inhibited, changes of two essential proteins ICAM-1 and VCAM-1 were examined, which were closely related to migration and invasion. The results showed that ICAM-1 and VCAM-1 were visibly decreased after inhibiting miR-190a-3p (Figure 3(d)).

RETRACTED

### 3.4. miR-190a-3p Negatively Regulates Its Target YOD1

In order to illustrate the mechanism of miR-190a-3p's effect on glioma, we first used TargetScan (V7.2) to predict the targets that interacted with miR-190a-3p. Among the candidate genes, YOD1 was selected for further study. The predicted interaction site of 3′UTR of target YOD1 to miR-190a-3p is shown in Figure 4(a). Meanwhile, according to the predicted interaction site of the 3′UTR of YOD1 with miR-190a-3p, dual-luciferase reporter plasmids were synthesized and cointroduced with miR-190a-3p mimics into glioma cells. The results are shown in Figure 4(b), indicating that YOD1 was indeed the target of miR-190a-3p. Next, we examined the level of YOD1 in glioma; it was shown that YOD1 was low-expressed in both glioma tissues and cells (Figure 4(c)). To investigate the relationship between the level of YOD1 and miR-190a-3p, we analyzed the included clinical samples and found that the level of YOD1 was negatively related to miR-190a-3p (Figure 4(d)). In addition, increased YOD1 expression was detected in glioma cells after the introduction of miR-190a-3p inhibitor (Figures 4(e) and 4(f)).

### 3.5. Silencing YOD1 Reverses the Effect of miR-190a-3p Inhibitor

For confirming the relationship between YOD1 and miR-190a-3p, we first designed shRNA to silence YOD1 expression, as shown in Figure 5(a). Next, we used CCK-8 and colony formation assays to confirm that sh-YOD1 could reverse the inhibited proliferation of glioma cells caused by miR-190a-3p inhibitor (Figures 5(b) and 5(c)). Besides, the silenced YOD1 alleviated the apoptosis induced by miR-190a-3p inhibitor as well as promoted migration and invasion of glioma cells to a certain extent (Figures 5(d)–5(f)). These results verified the negative relationship between miR-190a-3p and YOD1.

## 4. Discussion

Glioma is a malignant intracranial tumor. Nowadays, on a global scale, the treatment of this disease is still based on traditional treatment, such as surgery-assisted radiotherapy or chemotherapy. However, the prognosis for patients undergoing surgery is poor, mainly because this tumor is invasive and it is difficult to completely remove the lesion after surgery [20]. At the same time, the occurrence and development of glioma are a comprehensive process involving multiple factors, genes, and molecules; the specific pathogenesis of the disease is still unclear, so glioma is still a malignant tumor with poor prognosis and easy recurrence [21]. In recent years, more and more scholars focused their research on molecular-targeted therapy and proposed many new treatment schemes for various tumors.

RETRACTED

Recent studies on glioma have found that miRNAs play an essential part in the progress or apoptosis of tumor cells via controlling the expression of some key genes, such as p53 [22, 23]. Research has found that the upregulated miRNAs in glioma cells include the miR-183 [24], miR-21 [25], and miR-221 [26], while the downregulated miRNAs include miR-122 [27], miR-145 [28], and miR-26a [29]. Ding et al. found that in SHG-44 cell line, when the level of intracellular miR-122 was increased, the level of caspase9/3 was significantly increased, as well as the apoptosis rate. Further analyzing the target genes of miR-122 found that it may regulate apoptosis in glioma cells by inhibiting the expression of endogenous Bcl-w protein, which implied that the increased miR-122 inhibits the expression of endogenous Bcl-w and thus regulating the apoptosis process of glioma cells, playing an essential part in the appearance and progress of glioma [27]. Chen et al. validated that miR-105, miR-16, and miR-195 are low-expressed in U251, U87, SHG44, and MO59K cell lines. These three miRNAs could inhibit the metastasis of glioma cells and induced cell apoptosis. Besides, they combine with and inhibit the expression of SALL4, implying that these three miRNAs take part in the progress of glioma by regulating SALL4 [30].

In this paper, we explored the function of miR-190a-3p and its target YOD1 in glioma. The expression of miR-190a-3p was found markedly upregulated in glioma, whereas the level of YOD1 was markedly decreased. Suppression of miR-190a-3p restrained the progress and accelerated apoptosis of glioma cells. In addition, the expression of miR-190a-3p is negatively related to the expression of its target gene YOD1, and miR-190a-3p negatively controls the expression of YOD1. The rescue assay further validated the relationship between miR-190a-3p and YOD1, as well as their role in the progression of glioma.

Our research demonstrated that miR-190a-3p could promote the proliferation and migration of glioma through its target gene YOD1. The progression of glioma could be suppressed by inhibiting miR-190a-3p or overexpressing its target YOD1. This inhibition effect might be achieved by promoting cell apoptosis of glioma. In the future, we will continue to investigate the mechanism of apoptosis initiation after inhibition of miR-190a-3p. Besides, the in vivo experiments also need to validate. In general, our findings provide a novel approach for molecular therapy of glioma that can attempt to inhibit the proliferation and metastasis of glioma by inhibiting the expression of miR-190a-3p.

## Figures and Tables

**Figure 1:** miR-190a-3p is high-expressed in glioma. (a) miR-190a-3p in normal and cancer tissues. (b) miR-190a-3p in glioma tissues of grade I+II and III+IV. (c) Comparison of overall survival rate of clinical samples with high and low expression of miR-190a-3p. (d) Relative level of miR-190a-3p in HEB and four different glioma cell lines. (e, f) The miR-190a-3p inhibitor was introduced into U87 and U251 cell lines, and GFP was used to verify the transfection efficiency. ^∗∗^*p* < 0.01. Scale bar = 100 *μ*m for (e).

RETRACTED

**Figure 2:** Low-expressed miR-190a-3p can suppress the proliferation of glioma and promote its apoptosis. (a, b) The influence of inhibiting miR-190a-3p on the growth of U87 and U251 cell lines was evaluated by CCK-8 and colony formation assays. (c, d) TUNEL assay (c) and Western blot (d) were conducted to evaluate the cell apoptosis after transfection of miR-190a-3p inhibitor. ^∗∗^*p* < 0.01. Scale bar = 50 *μ*m for (c).

**Figure 3:** Low-expressed miR-190a-3p can suppress the progression of glioma. (a) The degree of wound healing in the miR-190a-3p inhibitor group was visibly lower than that in the control group. (b, c) Cell migration and invasion ability of the miR-190a-3p inhibitor group were markedly weakened. (d) The expression of ICAM-1 and VCAM-1 decreased markedly after introducing miR-190a-3p inhibitor. ^∗∗^*p* < 0.01. Scale bar = 50 *μ*m for (a–c).

**Figure 4:** miR-190a-3p negatively regulates its target YOD1. (a) The predicted binding site of YOD 3′UTR and miR-190a-3p. (b) The luciferase activity significantly decreased after introducing miR-190a-3p inhibitor and WT 3′UTR of YOD1, while the MUT YOD1 3′UTR group had almost no change. (c) Relative expression of YOD1 in glioma cell lines and tissues. (d) Relative expression of miR-190a-3p and YOD1 in clinical sample tissues was negatively correlated. (e, f) After introducing miR-190a-3p inhibitor, the expression of YOD1 in U87 and U251 cell lines increased. ^∗∗^*p* < 0.01.

**Figure 5:** Silencing YOD1 can reverse the effect of miR-190a-3p inhibitor. (a) YOD1 was silenced after being transfected with sh-YOD1. (b, c) The suppression of cell proliferation caused by miR-190a-3p inhibitor could be relieved by silencing of YOD1. (d, e) After cotransfection with miR-190a-3p inhibitor and sh-YOD1, the apoptosis of cells was relieved, compared with the cotransfected miR-190a-3p inhibitor and sh-NC group. (f, g) Silencing YOD1 could improve the reduced metastasis capacity of glioma cells caused by miR-190a-3p inhibitor. ^∗^*p* < 0.05 and ^∗∗^*p* < 0.01 vs. miR-190a-3p inhibitor+sh-NC group, ^##^*p* <0.01 vs. miR-190a-3p inhibitor+sh-YOD1 group. Scale bar = 100 *μ*m for (d), (f), and (g).

RETRACTED

**Table 1:** RT-qPCR primer sequences.

Gene	Primer sequences (5′-3′)
miR-190a-3p	Forward 5′-CTAGGAGCTTCAGTAACGTTA-3′
	Reverse 5′-GAATTCGAATCGGTAACAGCT-5′
YOD1	Forward 5′-CTTTGAAGCCAAGTAGCTTC-3′
	Reverse 5′-AAGTCAGTTGVATGAGCTGA-3′
U6 snRNA	Forward 5′-CTGATCAGTGAGTAAGATG-3′
	Reverse 5′-ATCGAATATGCAGTGTCAG-3′
*β*-Actin	Forward 5′-ACTGTTATGATAGCATCGA-3′
	Reverse 5′-CATACTGCATCCTATCGAAT-3′

## Data Availability

All data generated or analyzed during this study are included in this published article.
